# Grammar System of TCFL Driven by Neural Network Technology

This article has been retracted.

**DOI:** 10.1155/2022/9800539

**Published:** 2022-06-29

**Authors:** Rui Xiao, Shengquan Luo

**Affiliations:** Faculty of Education, Southwest University, Chongqing 400715, China

## Abstract

With the economy's continued and stable growth, China's political and economic influence in the international community has grown, and more and more friends from all over the world are requesting to learn Chinese and visit China. The growth of information technology and curriculum integration has had a significant impact on TCFL (teaching Chinese as a foreign language). Facing the new situation will enable us to gain a fresh perspective on the current state of TCFL grammar system research. Through specific teaching practice, this paper verifies the effectiveness of teaching Chinese as a foreign language and cultural vocabulary. This paper proposes a grammar error correction scheme based on hybrid models—Transformer model and N-gram model—that dynamically combine the outputs of different neural modules to improve the model's ability to capture semantic information, with the goal of correcting Chinese grammar errors. Experiments show that the Transformer and N-gram model-based Chinese grammar error correction strategy performs well in the global effect, and the overall performance is the best in the detection and positioning levels. At the detection level, the model in this document has the highest error correction accuracy of 0.64 and the highest recall rate of 0.67. The results show that adding an attention mechanism to a grammatical error correction model can improve its computational efficiency.

## 1. Introduction

Since the founding of new China, TCFL (teaching Chinese as a foreign language) has a nearly half-century history. Chinese as a foreign language has progressed rapidly, with gratifying achievements in both theoretical research and teaching practice, as a result of the deepening of theoretical research and the enrichment of teaching experience. When it comes to learning a second language, grammar is essential. Teaching experience has shown that if you only learn the grammar of one language, you will not be able to learn that language well; however, if you want to learn a second language well, you must learn its grammar as well. An important sign is mastering the grammar of a second language [1]. TCFL now faces new challenges as a result of the new situation. The three main tasks before us are textbooks, teachers, and teaching methods, all of which are directly related to the quality of teaching and the success or failure of Chinese international promotion.

The characteristics of the information society have posed new challenges to the traditional education in schools and put forward new ideas for talent cultivation for education and teaching, which are organically integrated with the curriculum. Lin et al. think that information technology in integration should be able to guide, strengthen, and expand learning objectives, and technology as an integration tool should play the same role as other learning tools [2]. Under the background of actively promoting quality-oriented education and modernization and informatization of education, information technology must be for students to choose and analyze information services. Luo and Yang studied the integration of information technology and regional planning course, which is a college preparatory course, using the teaching methods such as the implementation of the planning scheme and the application, and thought that the teaching methods were participatory and experimental [3]. Han thinks that the integration mode can be divided into two categories: first is classroom teaching integration, and second is autonomous learning integration, as well as, specifically, online teaching, individual learning, and online discussion [4]. Shi and Yang made a comparative analysis of the teaching modes before and after the multimedia entered the newspaper class through application examples. The results showed that the role of multimedia in newspaper reading class surpassed other classes, not only helping teachers to complete a large number of teaching contents but also changing the boring atmosphere in the previous class [5]. Ahmad and Rao optimized and improved the experiential game model. Through this model, game designers can have a deeper understanding of the learning mechanism in games, highlight the factors that make games playable, and try to describe game-based learning from different levels, trying to integrate the teaching principles into the design of games [6]. White points out that grammar should focus on imparting a language skill from the perspective of language application rather than language knowledge from the perspective of linguistics and emphasizes sorting from the perspective of function [7]. From the perspective of textbook compilation, Chan puts forward the “Discovery Grammar Compilation Model,” which requires that the principles of autonomy, comprehensiveness, communication, and integrity should be followed [8].

The integration of information technology and TCFL grammar system can promote the computerization of TCFL education, including the sharing of TCFL platform, TCFL computerization, TCFL customization, and automation of management evaluation system. At the same time, information technology can provide unprecedented means for the design and implementation of TCFL grammar system, making it possible to implement personalized courses. Using the communication and speed of information technology, after-class feedback is more timely, students' learning effect is better, and teachers' guidance is more specific. This topic fully demonstrates the operability of the integration of information technology and Chinese as a foreign language, with a view to providing some ideas and teaching models for the application of information technology in Chinese as a foreign language classroom.

The innovation of this paper is summarized as follows:

1. Combining information technology theory with TCFL grammar system courses and characteristics, we can realize digital Chinese learning. The goal of integrating information technology with Chinese as a foreign language is to change the traditional teaching structure, create an ideal Chinese learning environment, and improve students' Chinese information literacy.
2. A grammar error correction scheme based on the combination of Transformer and N-gram model is implemented. Parallel corpus is obtained by preprocessing the training data, and it is used to train the grammar error correction model.

The full text is divided into five chapters, and the contents of each chapter are distributed as follows.

The first chapter introduces the research background and significance and then introduces the main work of this paper. The second chapter mainly introduces the related technologies of grammar error correction. The third chapter puts forward the concrete methods and implementation of this research. The fourth chapter verifies the superiority and feasibility of this research model. The fifth chapter is the summary of the full text.

## 2. Related Work

### 2.1. TCFL Grammar Research

TCFL grammar refers to the part about grammar in TCFL. Generally speaking, there are five different forms of annotation and grammar exercises in textbooks: reference grammar, grammar books or textbooks (including exercises) mainly used by students for self-study, classroom grammar teaching, teach grammar theory, and so forth.

It plays an important role in the construction and mastery of grammar in second language teaching. Therefore, the formation of grammar system has become the central theme and historic achievement of the discipline construction of second language teaching. Learning grammar is mainly about learning grammar knowledge, so as to understand the mother tongue reasonably and improve the language expression ability and logical thinking ability. The purpose of teaching Chinese grammar as a foreign language is to teach a language, that is, to teach a language by teaching grammar, and then to learn a language by learning grammar; that is, grammar teaching is a means and the fundamental purpose is to cultivate Chinese language ability and language communication ability.

Roig believes that TCFL grammar is not systematic but more “menu.” There is no “TCFL grammar system” but “TCFL grammar item list” [9]. Pan holds that the ordering principle of teaching grammar points depends on the degree of difficulty. Grammatical structures with low difficulty in teaching should appear earlier, and grammatical structures with high difficulty should appear later [10]. Lin suggested the following: “Based on the fact of Chinese grammar, we should use the grammar theory of ‘syntax, semantics and pragmatics' to perfect the construction of TCFL grammar system” [11]. According to Akkaya, there is no absolute order of all grammar points, but some grammar points are in order. The difficulty of grammar is not the absolute principle of ordering [12]. Guo and Yang further put forward clearly that the focus of grammar teaching should be on language use, and the explanation of grammar terms and rules is only a means of grammar teaching, and the goal of grammar teaching is to cultivate students' language use ability [13]. Garcia believes that we teach grammar rules, not grammar knowledge, so we are opposed to lecturing grammar in class [14]. On the contrary, we think that grammar teaching should be downplayed, and it is better to teach grammar without any trace. Let students master grammar rules unconsciously.

### 2.2. A Summary of the Research on Chinese Grammar Error Correction Methods

Compared with English, Chinese grammar is more complicated and flexible. Because there are no clear grammatical rules in Chinese, such as singular, plural, and word tense, its grammatical errors often involve implicit semantic analysis, which cannot be judged according to the form of words. Therefore, the most common mistakes made by Chinese learners in the process of learning Chinese are grammatical errors.

Bruton proposed a system combining manual language rules and N-gram model to detect Chinese grammatical errors in sentences [15]. Truscott adopts a simple-to-complex step-by-step error correction method, using language model to correct simple errors, and word-level Transformer model to correct complex errors [16]. He proposed a Chinese grammar error correction model based on Transformer enhanced architecture, which uses the dynamic residual structure combined with the outputs of different neural modules to enhance the ability of the model to capture semantic information [17]. Podymov used the sequence generation model of multilayer convolution and reordered the final generated results by using language model, and it became the first neural error correction model that surpassed statistical machine translation method [18]. Nakano used pattern matching method and sentence component analysis method to check, taking into account local and global grammatical restriction information [19]. Park et al. adopted the parallel structure of multiple models and used three kinds of models based on rules, statistics, and neural networks. First, they made low-level combination within categories to get category candidates and then made high-level combination of category candidates [20].

Many language learning and teaching systems based on artificial intelligence take corpus as one of their basic resources. Corpus is a basic database obtained by screening and marking a large number of target language texts. Sang-Keun exercises Chinese characters with a huge corpus and forms a maximum entropy model based on binary classification. The core idea is to treat all the characters in the text as a binary classification and to correct all the characters [21]. Bera et al. proposed applying the first-order probability summary learning method to error classification and performed comparison with some basic classifiers; it was found that it was indeed improved [22]; Skok et al. refined N-gram and POS-n-gram according to the traditional supervised submission, in which the frequency of N-gram was selected from a corpus to be referenced, and SVM (Support Vector Machine) was cited for training [23].

## 3. Methodology

### 3.1. Practice of Optimizing and Integrating Information Technology with TCFL

The development and dissemination of Chinese proficiency courses, Chinese teaching grammar courses, and general education courses have been aided by the grammar system and related research findings. Simultaneously, grammar teaching reference books that discuss the expression of grammar rules and the instruction of grammar teaching have appeared one after the other, gradually broadening and expanding the research on grammar system. When people began to study the media and other elements in the teaching process using the systematic process view, a new teaching concept emerged: relying on resources to promote effective teaching. As a foreign language, Chinese grammar must be productive, able to produce correct sentences and paragraphs according to learning rules. As a result, foreigner grammar instruction must have a clear focus, taking into account their difficulties and prejudices.

The network resources provided by information technology provide dynamic and continuous teaching materials and extracurricular learning resources for TCFL. Teachers can boldly introduce network resources into the classroom or use multimedia teaching materials and make full use of rich Internet resources to make the teaching materials vivid and easy to understand. By showing the teaching process to students through multimedia, the knowledge capacity of teaching materials is expanded, and Chinese culture is skillfully integrated. This not only enriches the contents of textbooks but also broadens students' horizons, makes them love Chinese culture more, and enhances their interest and self-confidence in learning Chinese.

Teachers' leading role in inquiry-based teaching is primarily manifested in the use of various information technologies to create Chinese situations, pose inquiry questions, and then guide and monitor students' Chinese inquiry activities. We should use multimedia to create situations in teaching from the beginning of grammar to the end, so that students can learn and apply grammar in real-life situations. Students can unconsciously say sentences containing grammatical points in the situation if flash animation or pictures are used for demonstration when importing. In practice, multimedia can be used to create a communication environment where students can practice their grammar. Teachers can demonstrate handwriting multiple times in class or allow students to practice according to time after class, which not only saves time for teachers who would otherwise have to repeat it in class but also helps students practice and remember it.

With the difficulty of TCFL, the mastery of cultural vocabulary is directly related to international students' understanding of Chinese culture and will further affect their communicative competence and language ability. In order to improve foreign students' cultural vocabulary level and communication level, we try to apply mind mapping to TCFL, as well as the differences of teaching effects between mind mapping and Chinese teaching, such as foreign languages and traditional teaching mode, in order to explore which method is more conducive to promoting international students to learn cultural vocabulary. In order to better apply mind mapping to TCFL, we have designed new mind mapping teaching courses and mind mapping application review courses. The instructional design is shown in Figure 1.

Because international students have little contact and understanding of mind maps, the content of the text is unfamiliar to international students. Therefore, when we teach new courses, we make rational use of blackboards and use colored chalk to teach and guide demonstrations. Therefore, the mind maps that students can understand are understandable, so international students can draw the knowledge map of mind maps in class. After class, we interviewed international students and found that many international students expect to use mind mapping in future courses. In the foreign language course of Chinese culture, students will be exposed to the basic knowledge of Chinese culture and the differences between Chinese and foreign cultures. Teachers can use various multimedia resources and media to present cultural teaching content, stimulate students' interest, and create a cultural atmosphere. When explaining, we should make use of the contrast between Chinese and foreign cultures to help students understand the basic knowledge of Chinese culture. The cultural discussion class of Accepting Chinese as a Foreign Language mainly includes the following links, as shown in Figure 2.

Information technology is being used in conjunction with cultural discussion courses, and the inquiry teaching mode is becoming more popular. Students study textbooks independently, use the Internet, libraries, newspapers, and magazines to obtain relevant information, and use all kinds of communication tools, information technology, and learning resources to fully explore the cultural charm of Chinese people. In class, discuss and share the results of your investigation. At any time, teachers will guide and monitor students' discussion and inquiry activities. Finally, summarize the comments and bring up the issue of cultural expansion so that students can continue to communicate outside of class by using the network platform.

The use of multimedia and other technological tools to teach grammar has yielded impressive results. Use concise and vivid formulas or tables to explain grammatical structure. Use images, animations, and other visual aids to create vivid, intuitive, and easy-to-understand concrete situations when explaining semantics and pragmatics. Teachers can now use information technology to provide real-life situations to their students, fully and thoroughly mobilizing their senses, improving learning efficiency, and breaking the monotony of grammar instruction. For example, in conjunction practice, teachers can show students various videos or pictures, have them practice according to the pictures, and then give them some sentences and words to do substitution exercises to help them understand and remember more.

### 3.2. Research on TCFL Grammar Error Correction Model

Different from English, Chinese is an ideographic character, its form has not changed according to the rules, there is no prescribed contrast between its words and syntactic elements [14], and no clear words are given in writing. It is difficult for foreign students to use their native language habits to learn Chinese correctly. In addition, under the influence of the mother tongue environment, it is difficult to accurately identify and correct grammatical errors. However, rules-level errors such as grammar, phrase placement, and word structure have become the most common types of errors. Therefore, the Chinese grammar error correction system becomes very important.

According to the rules of the language used by people, the output of the corpus is all words arranged in time series, so the following mathematical model can be abstracted. Let a sentence be a string sequence, and the words in *w*_1_, *w*_2_,…, *w*_*L*_ are all generated in chronological order. The language model calculation formula is as follows:

(1) $$\begin{array}{c} P\left(w_{1},w_{2},\cdots ,w_{T}\right)=\prod_{t=1}^{T}P\left(w_{t}|w_{1},w_{2},\cdots ,w_{t-1}\right). \end{array}$$

*P*(*w*_1_) is the ratio of the number of times *w*_1_ appears on the training set to the total number of times in the training set.

Transformer model is a sequence generation model encoder based on multihead attention mechanism (responsible for encoding input text into high-dimensional implicit semantic vector, and the decoder decodes the implicit semantic vector according to the output of the previous step as the output vector of the current step. The output vector of each step corresponds to one word, and the final output sentence is obtained by combining the output words of all steps.

The features of words or sentences in each coding layer learned by Transformer model may have different semantics; that is, they have learned features with hierarchical structure. For example, the top coding layer may represent the most intuitive meaning of a sentence, while other layers may represent the most intuitive meaning of a sentence. You can learn the deeper language features of sentences. Attention of each attention layer takes the dot product of rank, as shown in the following formula:

(2) $$\begin{array}{c} Att\left(Q,K,V\right)=\text{soft}\max\left(\frac{QK^{T}}{\sqrt{d_{k}}}\right)V, \end{array}$$

(3) $$\begin{array}{c} \text{Multi\_Head}=\left[Att_{1},Att_{2},\cdots ,Att_{h}\right]. \end{array}$$

In formula (2), *Q*, *K*, *V* represent the query matrix, key value matrix, and real value matrix of attention layer, respectively; *d*_*k*_ is the third dimension size of the embedding layer of the mold; Multi_Head is the splicing of multiple attentions.

According to the calculation range of the system, the attention mechanism can be divided into local calculation and global calculation. This paper mainly uses the soft Attention part of global calculation to identify and deal with language errors. Define the weight factor *α*_*ij*_, and the calculation formula is as follows:

(4) $$\begin{array}{c} \alpha_{ij}=\frac{\exp\left(e_{ij}\right)}{\sum_{k=1}^{T_{x}}\exp\left(e_{ik}\right)}, \end{array}$$

(5) $$\begin{array}{c} e_{ij}=\alpha \left(s_{i-1},h_{j}\right). \end{array}$$

We accumulate the outputs of all neural modules as the final output, as shown in Figure 3, so that the gradient of loss function will not disappear with the increase of model depth. Using the output of the last neural module directly as the general output of encoder or decoder may lead to the loss of some semantic information.

This dynamic residual structure can be applied to the encoder or decoder of Transformer model, which can not only help the model capture richer semantic information but also reduce the gradient attenuation caused by too deep modeling and make the network better trained.

At present, the N-gram model is the most widely used and well-operated language model, with simple structure and good prediction ability. The core element of the N-gram method is to use the detected text to follow the pattern of bytes to implement the moving window operation with the specification of *N*, thus forming a byte fragment sequence with the length of *N*, and each byte fragment is named gram [14].

In the N-gram language model, it is assumed that the occurrence of the *n* word is only related to the first *n* − 1 word and has nothing to do with all other words. Therefore, the probability of this sentence is equal to the product of the probabilities of each word's occurrence, and the probability can be obtained by counting the number of common occurrences of words in the corpus.

For the N-gram language model, let *S* represent a sentence with actual meaning, and it is composed of a series of *n* components *w*_1_, *w*_2_,…, *w*_*n*_ listed in a specified order, which can be words or phrases. The probability distribution is *P*(*S*):

(6) $$\begin{array}{c} P\left(S\right)=P\left(w_{1},w_{2},\cdots ,w_{n}\right). \end{array}$$

From the above conditional probability formula, it can be concluded that the probability of occurrence of *S* statement sequence is equal to the product of conditional probabilities of occurrence of all words in the sequence.

After the value of *N* is determined, the next step is to build the model. Before building the model, it is necessary to build a suitable corpus to practice the model. Bigram model probability *P*(*S*) is expressed as

(7) $$\begin{array}{c} P\left(S\right)=P\left(W_{n}|W_{1},W_{2},\cdots ,W_{n-1}\right)=\frac{c\left(w_{1}w_{2},\cdots ,w_{n}\right)}{c\left(w_{1}w_{2},\cdots ,w_{n-1}\right)}. \end{array}$$

In the above formula, *c*(*w*_1_, *w*_2_,…, *w*_*n*_) represents the number of times *W*_1_, *W*_2_,…, *W*_*n*_ appears in the dataset. According to the above formula, its probability solution formula can be converted into

(8) $$\begin{array}{c} P\left(S\right)=P\left(W_{1}\right)\cdot \frac{c\left(w_{1}w_{2}\right)}{c\left(w_{1}\right)}\cdot \frac{c\left(w_{2}w_{3}\right)}{c\left(w_{2}\right)}\cdots \frac{c\left(w_{n-1}w_{n}\right)}{c\left(w_{n-1}\right)}. \end{array}$$

The low-order N-gram model is used to linearly interpolate the high-order N-gram model. When there is not enough data to estimate the probability of the high-order model, the low-order model can generally provide valuable information to evaluate the probability estimation of the high-order model. The detailed formula is shown as follows:

(9) $$\begin{array}{c} P\left(w_{n}|w_{n-1},\cdots ,w_{n-i+1}\right)=\lambda_{1}P\left(w_{n-1}|w_{n-1},\cdots ,w_{n-i+1}\right)+\lambda_{2}P\left(w_{n-1}|w_{n-1},\cdots ,w_{n-i+1}\right)+\cdots +\lambda_{i}P\left(w_{n}\right). \end{array}$$

The probability formula of *N*=1,2,3,4,5 combination model obtained by linear interpolation smoothing algorithm is as follows:

(10) $$\begin{array}{c} P\left(S\right)=\prod_{i=1}\lambda_{N}p\left(w_{i}|w_{i-N+1}^{i-1}\right). \end{array}$$

The syntax error correction module of this model is based on a variety of syntax error correction models to form a parallel structure. It mainly integrates the traditional syntax error correction model and depth model, uses the low-level model for routine error correction, leaves the high-level error correction for depth, and combines the neural network model to correct syntax errors. The models can run independently and have no dependence on each other. In addition, each model can preprocess data, train, and predict independently. The system error correction process is shown in Figure 4.

After the user completes the grammar correction, if the user is not satisfied with the correction result, it will be returned to the system. You will be prompted to focus on the information in the article. System bug fixes will be updated and modified regularly by administrators, and the model will be set according to the threshold. At the same time, the text information modification database obtained from the feedback will also be used as one of the corpus resources to participate in the grammar error correction operation.

## 4. Experiment and Results

### 4.1. Analysis of Teaching Method Effect

Compared with the traditional educational mode and media, multimedia technology and network technology brought by information technology have many advantages. They open our classroom, broaden our horizons, enliven the classroom atmosphere, and provide a variety of ways and choices. The closed and unique traditional education mode is beneficial to arouse students' enthusiasm and improve the quality of TCFL. The use of information technology is a means, not an end. Even advanced tools cannot replace teachers' teaching and students' learning. However, the varied and elegant teaching materials will not be more impressive and effective than the rich classroom contents.

As an effective teaching method, we applied mind mapping to TCFL practice and conducted a four-month empirical study on the effectiveness of mind mapping in teaching Chinese as a foreign language cultural vocabulary. The results in Table 1 show that, among the 40 international students surveyed, 32 international students think mind mapping works well in class, and 8 international students think traditional class works better.

Through a semester-long experimental study, the authors summarize the proportion of international students who have reached different levels in the two exams. Through a comparative analysis of three-exam data, it is found that, from the cognitive level, compared with the previous level tests, the proportion of international students in cultural words, institutional cultural words, behavioral cultural words, psychological cultural words, and spiritual cultural words decreases, while the proportion of idioms increases, which shows that mind mapping has a certain influence on foreign students' understanding of cultural words. See Figure 5.

In terms of proficiency, compared with the previous placement test, after using mind map teaching, international students are more proficient in material cultural vocabulary, institutional cultural vocabulary, behavioral cultural vocabulary, cultural vocabulary, and psychological, spiritual, and cultural vocabulary and idioms. See Figure 6.

Through the comparative analysis of the data from the two tests, the application of mind mapping teaching method in TCFL class can help foreign students improve their vocabulary. Most students have mastered what they have learned. Compared with the previous teaching methods, the gamification classroom has certain advantages in cultivating students' interest in learning Chinese, expression ability, cooperation ability, and problem-solving ability. Teachers also said that, after this teaching practice, they have a deep understanding of gamification learning, and they will continue to study and apply the idea of gamification to future TCFL.

The integration of information technology and Chinese as a foreign language has changed the traditional dual mode of teachers and students in Chinese as a foreign language classroom, and any information education technology cannot replace the leading role of teachers. Teachers' wonderful deduction can turn simple classroom into wonderful classroom. Teaching Chinese as a foreign language is not only a process of imparting Chinese knowledge but also a process of spreading Chinese culture. Teachers should make full use of the unique potential of modern information technology, show their own teaching style, create an environment suitable for students, and organize, guide, help and supervise them, starting from the subject or teaching content and students' emotional characteristics.

### 4.2. Analysis of Grammatical Error Correction Model

In this chapter, BIO labeling is used to transform the joint labeling in the original labeling problem.

The meanings of labels in BIO annotations are as follows: *B* (begin), *I* (in), *O* (out), where “*B*-*X*” indicates that this element belongs to the *X* part of the speech and is located at the beginning of the segment; “*I*-*X*” means that the element belongs to the grammar part and is in the middle of the segment; “*O*” means that the element does not belong to any syntax part.

The first experiment is to use the model to evaluate the error labels set in this paper. The experimental data are shown in Table 2.

From the above experiments, it can be seen that the accuracy of the wrong words is higher than that of other types of errors, and the overall performance of all types of errors is relatively average in terms of recall rate and *F* value, with little difference.

In the second experiment, under the same experimental conditions, the error correction model constructed in this chapter is compared with other different grammatical error correction models, and the detection level and positioning level are, respectively, compared. The results of the experimental data are shown in Figures 7 and 8.

From the above experimental data, it can be seen that the Chinese grammar error correction strategy based on Transformer and N-gram model performs well in the overall effect, and the overall performance is the best in the detection level and detection position. The model in this document has the highest error correction accuracy of 0.64 and the recall rate of 0.67 at the detection level. Compared with CNN model, the error correction strategy based on Transformer and N-gram model can capture long-distance and short-distance bidirectional information, and CNN layer can directly use information data. The model in this paper is based on character level research. Although it has a strong long-term memory function, the lack of word placement information leads to the decline of placement level effect. Therefore, in the future work, we will continue to explore adding external functions to improve the error correction performance of the model. At the same time, we also analyze the impact of data enhancement methods, including the impact on *F* values of six specific error types in the test set, as shown in Figure 9.

As can be seen from Figure 9, after using the data enhancement method, nouns, symbols, word order, and four other types of errors are obviously improved, but the errors are not effectively improved. Therefore, the data enhancement strategy should be able to increase the number of different types of errors year by year.

## 5. Conclusions

Faced with the onslaught of global Chinese fever and the need for new teaching methods, the investigation of the TCFL grammar system should help to clarify the current state of grammar teaching by reexamining the TCFL system. A successful integration case is chosen to verify and give feedback on the integration model research based on the research of information technology integration model and TCFL grammar system. According to the findings, using mind mapping in TCFL practice increased foreign students' interest in learning Chinese and Chinese culture, as well as their enthusiasm for participating in classroom interaction. The combined Transformer and N-gram model is used to correct Chinese grammar errors, and Chinese word segmentation technology is used. The model streamlines the process by integrating error detection and correction. Experiments show that the Transformer and N-gram model-based Chinese grammar error correction strategy performs well in the global effect, and the overall performance is best in the detection and positioning levels. At the detection level, the model in this paper has the highest error correction accuracy of 0.64 and the highest recall rate of 0.67. The feasibility of using the Transformer and N-gram model to correct Chinese grammar errors has been established, and this model can also be applied to other tasks.

## Figures and Tables

**Figure 1:** Teaching design drawing.

**Figure 2:** Elements of the teaching mode of receptive cultural discussion class.

**Figure 3:** Dynamic residual structure.

**Figure 4:** Chinese grammar error correction model design.

**Figure 5:** Three tests of foreign students' ignorance.

**Figure 6:** Test the proficiency of foreign students three times.

**Figure 7:** Comparison at the detection level.

**Figure 8:** Comparison at the positioning level.

**Figure 9:** Influence of using data enhancement method on different error types.

**Table 1:** Comparison between traditional classroom and mind map classroom effect.

Nationality	Overall number of people	Traditional classroom		Mind mapping classroom	
		Total number of people	Proportion (%)	Total number of people	Proportion (%)
Russia	26	5	19.2	21	80.8
Britain	9	2	22.2	7	77.8
Japan	3	1	33.3	2	66.7
Pakistan	2	0	0	2	100
Total	40	8	20	32	80

**Table 2:** Error label evaluation experiment.

Label	Precision	Recall	*F* value
*B*-*R*	0.22	0.13	0.19
*I*-*R*	0.24	0.05	0.15
*B*-*M*	0.15	0.16	0.22
*I*-*M*	0.00	0.00	0.00
*B*-*S*	0.23	0.14	0.21
*I*-*S*	0.28	0.11	0.23

## Data Availability

The data used to support the findings of this study are available from the corresponding author upon request.
